# Research on Information Visualization Graphic Design Teaching Based on DBN Algorithm

**DOI:** 10.1155/2021/3355030

**Published:** 2021-09-28

**Authors:** Manjun Xue

**Affiliations:** School of Architectural and Artistic Design, Henan Polytechnic University, Jiaozuo 454000, China

## Abstract

With the advent of the era of big data, how to quickly obtain effective information and efficiently disseminate information technology has become the most popular topic. Studies have shown that the ability of the human brain to process data and information is unmatched by machines, and the processing of graphics is tens of thousands of times faster than that of words. Based on the deep belief network (DBN) algorithm, this paper studies the technology of information visualization graphic design teaching application. Firstly, the structure of the deep belief network is analysed to explore its technical application in graphic information reconstruction. It is concluded that the DBN algorithm can be used to deal with the problems of classification, regression, dimension calculation, feature point acquisition, accuracy calculation, and so on in machine learning training. Then, the deformation technology of graphic local design is studied based on the DBN algorithm to construct the visual teaching platform and analyse the technical research results of this algorithm in information graphic design. The results show that the DBN algorithm can quickly solve the problem of processing complex features in graphics, change the local deformation design of the original graphics to form new feature point data and add it to the teaching platform, and improve the ability of model fast learning and training, optimizing the operation efficiency of the teaching platform.

## 1. Introduction

With the rapid development of big data 5G era, today's media society has dual tasks of information transmission and processing [1]. According to many scholars, the speed and efficiency of human brain processing information is very high. Among them, the information processing and processing of pictures and graphics are tens of thousands of times faster than that of words, so if we want to realize machine learning training, we first start with graphics and images [2, 3]. Due to the increasing demand for information graphic design, more and more people are willing to study information graphic design [4]. The basic idea of this major is to realize the course of graphic visualization based on data information. In the teaching design, we need to study the visual graphic display of data information acquisition, capture, screening, logical structure, and so on [5, 6].

In the traditional teaching mode, we should first cultivate students to be able to independently collect data, knowledge, information, and other elements about the subject content [7]. Then, the course training is used to enable students to learn the captured data information quickly and systematically. Deep learning, also known as the artificial neural network, can build a variety of machine models to replace human training and learning process [8, 9]. At present, the deep learning algorithm is developing rapidly in artificial intelligence, intelligent recognition, simulation modelling, image processing, and other fields. Among them, genetic neural network, convolution neural network, cyclic neural network, deep belief neural network, and other algorithm models are constantly applied in various fields [10]. In order to improve the defects of traditional information visualization graphic design teaching, such as inability to handle a large number of data information, low transmission rate, and inaccurate output data results [11]. We use the deep belief algorithm (DBN) in deep learning to optimize the teaching of information visualization graphic design. In order to solve the problem of fast and automatic learning in machine learning, the deep belief network is a fast learning and training algorithm of DBN [12]. By analysing the DBN algorithm model, this paper develops a new direction of the deep learning algorithm and applies this technology to various fields [13]. The DBN algorithm can carry out preprocessing, that is, fusing feature points to improve the structure of complex data nodes and improve the accuracy and quality of data input in the model. According to the neural network optimization, the model parameter variables are formed [14, 15].

This paper is divided into three parts. The first part is a brief introduction of the development of the deep belief algorithm in deep learning and the basic idea of information visualization graphic design teaching. Thus, a teaching research content of information visualization graphic design based on the DBN algorithm is proposed. The second part is related work about discussions on some related papers in this field. The third part is the graphic processing technology in information graphic design by using the DBN network algorithm structure. This paper mainly focuses on deep belief network structure technology and graphic reconstruction algorithm in the teaching platform. Then, the construction of the visual teaching platform for information graphic design is studied. This paper analyses the pattern of graphics classification and processing in teaching. The fourth part is the result analysis of the teaching research of information visualization graphic design based on the DBN algorithm. Firstly, the results of this algorithm in the reconstruction of information graphics are analysed. Finally, the research results of the deformation processing technology model of information graphics design using the DBN algorithm are analysed. The final part is the conclusion to show some important findings and suggestions.

## 2. Related Work

Information graphic design needs to display the acquired data and information graphically. In this process, it needs to meet the requirements of clarity, accuracy, and readability of graphic information [16]. Therefore, we need to choose the logical relationship suitable for this kind of professional nature in teaching design, process the complex and miscellaneous data information, and sort and classify the information [17]. In traditional teaching, students need to repeat the training and learning of information graphic design for many times. In the machine model, it is more necessary to make the teaching model be able to process the information data according to the thinking mode of the human brain to form the graphic transformation [18]. To complete the design of the whole teaching model, we first need to study and analyse the DBN algorithm and then use the visual construction tools to form the association between graphics and information. The information is automatically generated into the graphic data in the teaching model [19].

With the development of human brain science and computer science, the idea of the deep learning algorithm is gradually improved [20]. The technology of the artificial neural network training model is gradually concerned by researchers. In the field of education and teaching, the main technology is to transform the form of the basic neural network into deep learning training. Some schools have used the deep belief algorithm to optimize the cognitive structure, but the effect is not ideal. The reason is that the teaching mode pays too much attention to mechanical learning, which cannot give full play to students' innovation ability.

With the development of the deep learning algorithm, this algorithm is gradually combined with artificial intelligence devices [21]. It is mainly reflected in the deep learning of the DBN algorithm and backpropagation neural network combined with optimization, forming the ability to analyse the handwriting similarity and deal with fuzzy picture handwriting and other functions. In this experiment, they found that the neural network based on the DBN algorithm can accurately identify time parameters and improve the recognition efficiency and accuracy of the model.

According to the neural network algorithm and the case, scientists put forward a neural network structure optimized by the genetic algorithm [22]. This neural network structure is representative in human recognition, speech processing, image data analysis, and other fields. Subsequently, genetic algorithm optimization is combined with the deep belief neural network structure, and the main research direction is to apply this algorithm to solve the problem of incomplete text information. In addition, the text information is classified first, and the optimized DBN algorithm can recognize the wrong words in the case of a large number of missing text information.

The development of the deep learning algorithm is also at the forefront of the world [23]. Many researchers mainly analyse the performance of the deep learning algorithm and shallow neural network algorithm in the research of digital recognition [24–28]. Subsequently, it is confirmed that the deep belief network has great applicability and high efficiency. In the field of information graphics design, the model is built based on the DBN algorithm [29]. Experiments show that this algorithm can improve the accuracy of the model to express the meaning of abstract information data and can also quickly process graphic information and effectively classify information [30]. To sum up, this paper analyses the development trend of deep belief network technology in many countries. We use this algorithm to build the information visualization graphic design teaching model.

## 3. Research on Information Visualization Graphic Design Technology and Teaching Platform Design Based on DBN Algorithm

### 3.1. Research on Information Graphic Design Reconstruction Technology Based on DBN Algorithm

DBN algorithm is based on the development of artificial neural network optimization iteration, mainly using the biological neural network structure and shallow neural network structure basic idea to generate the probability calculation model. The distribution range of variable parameters in the sample data is calculated so that the weight value in the network structure can calculate the maximum probability of learning and training output data. The main function is to improve the accuracy of the training model and classification function, which can express the abstract meaning of information. The basic principle of this algorithm is to combine the superposition of RBM with the backpropagation neural network to form a deep learning supervision algorithm. In the process of model training, RBM can be trained from high to low to achieve the purpose of machine training. In the pretraining, the initial data of the structure variables of the supervisory layer neural network is set first, and then, the parameters of the variables of the model combined with the backpropagation neural network structure are slightly adjusted. Therefore, in the DBN algorithm structure, there is no other neural network structure calculation data gradient disappear phenomenon. It improves the accuracy and efficiency of the information visualization graphic design teaching model. The structure of the deep belief network is shown in Figure 1.

In the process of RBM, the complexity of data needs to be classified and planned. When the original BM structure of the Boltzmann machine is faced with complex data, the training time will be longer, which is not conducive to the training efficiency of the model. In order to improve this situation, the RBM structure is shown in Figure 2.

In the DBN algorithm structure, the input level and the fading level do not affect each other, but are formed by multiple RBMs and supervisors. There are two steps: no deep learning, supervised learning and training, and supervised microadjustment. In RBM hierarchy, the initial state needs to be assigned:

(1) $$\begin{array}{c} E=\left(v,h\;|\;\theta \right)=-\left(\sum_{v}w_{v}v_{t}h_{j}+\sum_{t}b_{t}v_{t}+\sum_{j}c_{j}h_{j}\right). \end{array}$$

One is composed of the weight value and connection node. The rest is formed by numerical calculation of the node offset position and input variable parameter dimension. Each variable corresponds to a state mode, and the smaller the state energy is, the more stable the whole model is. After the parameter variables are determined, the probability distribution of the network structure is calculated as follows:

(2) $$\begin{array}{c} p_{\theta }\left(v,h\right)=\frac{1}{Z\left(\theta \right)}e^{-E\left(v,h|\theta \right)},\\ Z\left(\theta \right)=\sum_{v,h}e^{-E\left(v,h|\theta \right)}. \end{array}$$

From the above formula, it can be determined that the state between the initial state and the node level is formed independently. The activation probability of each layer is as follows:

(3) $$\begin{array}{c} P\left(h_{i}=1\;|\;v\right)=\sigma \left(\sum_{j=1}^{m}w_{ij}\times v_{j}+c_{i}\right),\\ \sigma \left(x\right)=\frac{1}{1+\exp\left(-x\right)}. \end{array}$$

The above formula contains the activation function. When the state of the fade layer is determined, the activation functions are also independent of each other:

(4) $$\begin{array}{c} P\left(v_{i}=1\;|\;h\right)=\sigma \left(\sum_{i=1}^{n}w_{ij}\times h_{j}+b_{i}\right). \end{array}$$

Through the analysis of the RBM function, the DBN algorithm can be used to deal with classification, regression, dimension calculation, time sequencing, feature point acquisition, accuracy calculation, and other problems in machine learning training.

The experimental results show that there is no gradient reduction in the experimental data calculated by the DBN algorithm, which increases the effectiveness of training effect. In the process of model supervision training, it can effectively solve the problem of prolonged training time.

In this paper, we need to analyse and process the graphics in the teaching model and use data acquisition to build the graphics reconstruction system. The work content of data acquisition is to store and filter the information data obtained from measurement. Then, the information graphic data is transmitted to the graphic reconstruction system. The graphic design will be displayed on the machine through the reconstruction algorithm. By normalizing the nonlinear relationship between the distribution of parameters and variables, the approximate model formula is obtained as follows:

(5) $$\begin{array}{c} C=S\times G. \end{array}$$

The DBN algorithm is introduced into analytic layer calculation in graphic design image reconstruction calculation. Only the constant value of the variable is considered, and the sensitivity of the matrix does not need to be solved. The DBN algorithm is used to construct the nonlinear relationship between the output data and the input data. Finally, the gray value of the image can be obtained by detection. We will introduce the DBN algorithm to analyse the performance of the ordinary reconstruction system. The contrast curve between the amount of data collected and the accurate gray value of graphics is shown in Figure 3.

It can be seen from the curve changes in the figure that, after the introduction of the DBN algorithm, with the increase of the number of data, the accuracy changes at a certain height and basically tends to be stable. It shows that the introduction of the DBN algorithm can improve the processing accuracy of graphic design and reconstruction technology.

In the DBN algorithm, each RBM process needs to be updated iteratively, and the range and direction of variable parameters are different after each update. Therefore, it is necessary to redefine the calculation range. If the selected range is relatively large, it is easy to reduce the accuracy. If the selection range is small, the convergence feedback speed will decrease. In order to solve this problem, we use the adaptive algorithm to update the parameters. By changing the range of continuous iterations and the output data of direction control in the RBM training process, the calculation formula is as follows:

(6) $$\begin{array}{c} \eta =\left\{\begin{array}{c} \alpha \eta^{\prime \prime }\Delta \theta_{t}+\Delta \theta_{t-1}>0,\\ \beta \eta^{\prime \prime }\Delta \theta_{t}+\Delta \theta_{t-1}<0. \end{array}\right) \end{array}$$

In the formula, the value range represents the increase and decrease coefficient of the variable. If the direction of the variable parameter range updated in each iteration is the same, the coefficient will increase; otherwise, it will decrease. After the introduction of the adaptive algorithm, the mechanism of variable parameter updating is changed:

(7) $$\begin{array}{c} W_{ij}=W_{ij}+\eta^{\prime \prime }{\left(v_{i}h_{j}\right)}_{\text{data}}-{\left(v_{i}h_{j}\right)}_{k},\\ a_{i}=a_{i}+\eta^{\prime \prime }{\left(v_{i}\right)}_{\text{data}}-{\left(v_{i}\right)}_{k},\\ b_{j}=b_{j}+\eta^{\prime \prime }{\left(h_{j}\right)}_{\text{data}}-{\left(h_{j}\right)}_{k}. \end{array}$$

The updated parameters can represent the output results of the adaptive algorithm, and the connection weight value can also represent the difference between the update direction and that before the algorithm was introduced. By adjusting the stable time to speed up the fine-tuning speed, it can show that there is the possibility of instability when the data difference changes. When the range decreases, the fine-tuning range will also decrease. Therefore, in the training and learning preprocessing stage, this algorithm can accurately find the optimal solution of the function that meets the parameter conditions. In the process of DBN fine-tuning, the BP algorithm is usually used to supervise and adjust the parameters according to the gradient direction of the objective function. However, the feedback speed of this algorithm is slow when it is close to the value of the objective function, which will lead to the increase of the whole training time. Therefore, we use quasi-Newton method instead of the BP algorithm to reduce the gradient, so as to speed up the training and learning speed of the DBN algorithm. The comparison of feedback speed curves of the quasi-Newton algorithm and BP algorithm in the comparison of objective function parameters is shown in Figure 4.

It can be seen from Figure 4 that the feedback rate close to the objective function value by using quasi-Newton algorithm is higher than that by using the BP algorithm.

The quasi-Newton algorithm uses the numerical value of parameter objective function and derivative calculation to construct an approximate matrix for information, which can solve the defect of increasing time in the face of a large number of data parameters and can also meet the reservation of feedback speed. The objective function formula of the quasi-Newton algorithm is defined as follows:

(8) $$\begin{array}{c} Fy=\frac{1}{n}\sum_{k=1}^{n}Y-Y^{2}. \end{array}$$

The gray value of output data and the predicted output result are defined, respectively, in the formula, that is to say, the error in the gray value of the reconstructed image. In the fine-tuning operation, the DBN weight numerical formula is adjusted as follows:

(9) $$\begin{array}{c} y_{k+1}=y_{k}+\alpha_{k}d_{k}. \end{array}$$

The formula defines the search range direction of the arbitrary number of iterations and uses the range parameter to get the objective function gradient and search direction of the optimal data solution:

(10) $$\begin{array}{c} g=△Fy,\\ a_{k}=\arg\underset{a}{\min}fy_{k}+\alpha d_{k}. \end{array}$$

Through the above calculation, the final output data matrix is as follows:

(11) $$\begin{array}{c} B_{k+1}=B_{k}+\frac{y_{k}y_{K}^{T}}{s_{k}^{T}y_{k}}-\frac{B_{k}s_{k}s_{k}^{T}B_{k}}{s_{k}^{T}B_{k}s_{k}}. \end{array}$$

Therefore, according to the above formula, we can use the DBN algorithm in the teaching model of information graphics design to get the reconstructed graphics for design. This algorithm can also improve the accuracy of the whole model graphic design and the running speed of the teaching model. Comparing the DBN algorithm with the traditional probability calculation, the DBN algorithm can reduce the long-time problem of complex information processing in probability calculation. The iterative updating of the DBN algorithm with the adaptive algorithm can speed up the fine-tuning speed and increase the stability when the data changes. These are the advantages that ordinary probability calculation does not exist.

### 3.2. Research on Local Deformation Technology and Teaching Platform Model of Information Visualization Graphic Design Based on DBN Algorithm

With the advent of the era of big data, how to deal with a large number of information data to obtain demand content and knowledge is becoming a concern. Accurate translation and understanding are the key problem we need to solve. In the design of information graphics, the first thing is to realize the function of visualization. Information visualization can be calculated from the transmission of information in ancient stone wall painting. With the development of science and technology and the support of information technology, we also push the information visualization graphic design to a climax. Graphics is a means to carry the meaning of information. People communicate and transmit information according to the visual perception of the eye. That is to say, the information is conveyed and expressed visually, and the information content is integrated and classified in the appropriate graphic design carrier. Therefore, in the establishment of the information graphics design teaching model, graphics should be transformed first. First of all, this paper studies the graphic deformation design. In graphic design transformation, the simplest way is to modify the shape and control the deformation process. However, the traditional deformation design will produce boundary aliasing. In order to improve this situation, we propose to use the DBN algorithm to optimize the local deformation of graphics.

Firstly, the feature point is defined as the local deformation center, and then, the position and influence factors of the feature range are calculated. Then, the new graphic design style is obtained by adding pixels to supplement the deformation area. The feature pixels are used as the input data of the DBN algorithm, and the deformation function is obtained after obtaining the local information. The DBN algorithm can accurately capture the style features of graphics:

(12) $$\begin{array}{c} P\left(h^{\left(k\right)}\right)=P\left(H,h^{\left(1\right)},h^{\left(2\right)},\ldots ,h^{\left(l\right)}\right). \end{array}$$

According to the formula, the original graph is defined as the basic feature data of the DBN graph, and the advanced feature points of different levels of the graph deformation area are obtained through training and learning. Then, the influencing factor coefficient variable is defined. The pixel value range of each region is also different. The following formula is used to calculate the pixel value range:

(13) $$\begin{array}{c} l\left(v\right)=\frac{d\left(v\right)}{s\left(v\right)}\times g\left(l\right). \end{array}$$

In order to ensure the stability of deformation efficiency, we build a DBN graphic deformation simulation platform in the experiment. After preprocessing the collected data, the control group and the experimental group were set up, respectively. The original image was taken as the control group, and the graphic design based on the DBN algorithm was taken as the experimental group. The changes of the two groups of figures are shown in Figure 5.

To sum up, the use of the DBN algorithm for graphic design optimization can effectively achieve local design changes and quickly extract image feature points and input them into the visualization platform as calculation data. Comparing the two images, the graphic design optimization after the DBN algorithm can change the local features for reclassification. Local feature points are applied to the elements of building a new graphic design. Among them, we compare the number of feature points processed by the DBN algorithm with the number of feature points of original graphics under the image definition and image factors, as shown in Figure 6.

It can be seen from Figure 6 that the graphic design deformation data after the introduction of the DBN algorithm can quickly obtain the feature point information in the state of low graphics clarity. It is more feasible than using the original drawing to construct the teaching model. The input processed by the DBN algorithm is added to the visual teaching platform, which is mainly developed by visual c++. The standard system interface is adopted, and the function module includes two parts: teaching manager system and student system. The core algorithm of the teaching platform uses space technology to store the graphic design scheme and uses cloud data to automatically allocate and calibrate the acquired information data. The feature image processed by the DBN algorithm is stored by using the linear coordinate 3D space processing of the least square method. Finally, the new data of the graphic design can be extracted at any time in the teaching model.

## 4. Results Analysis of Information Visualization Graphic Design Technology and Teaching Platform Design Based on DBN Algorithm

### 4.1. Analysis of Research Results of Information Graphic Design and Reconstruction Technology Based on DBN Algorithm

In this paper, the DBN algorithm is used to realize the research of information graphic design reconfiguration technology. The grid of the source data graph is separated by the network structure, and a certain range threshold is set for the graph pixels. The gray value of the control pixel is 255, and the unified setting greater than the pixel range is 0. Finally, the original image is mapped to the reconstructed image after processing, and the gray image obtained is shown in Figure 7.

It can be seen from the above gray coefficients that the DBN algorithm can accurately classify the pixels that meet the requirements. The unified setting of the gray coefficient can simplify the problem that complex graphics cannot deal with in graphic design. In the process of image reconstruction, we analyse the effect according to the image correlation coefficient and image error. The larger the correlation coefficient is, the smaller the error value is, which proves that the effect of image reconstruction is more feasible and efficient. The contrast coefficient between the DBN algorithm and traditional algorithm is shown in Figure 8.

According to the comparison curve in the figure, the reconstructed graph of the DBN algorithm is obviously better than that of the traditional algorithm and has higher conversion effect. Compared with the original way to obtain feature points, the reconstruction system under the DBN algorithm can optimize graphic features and accurately capture the differences in similar graphic designs. Finally, a large number of different data obtained are unified for image reconstruction, which can provide a new design scheme for information visualization graphic design. The DBN algorithm also has faster training and learning speed than the traditional algorithm in the fine-tuning stage, which improves the speed of graphic design training in the teaching model. That is to say, when the teaching model carries out real-time information transmission, it can generate the graphic design scheme to express the information content faster.

### 4.2. Analysis of Local Deformation Technology in Information Visualization Graphic Design Based on DBN Algorithm

In order to prove that the local deformation technology of information visualization graphic design based on the DBN algorithm can help the teaching model increase the graphic design data and reduce the graphic preprocessing error, in the experiment, we will get the information first for content analysis, and then, after preprocessing normalization operation, the image is divided into the deformable region and original region. Compared with the original image, we can see that the deformation process using the DBN algorithm is ideal, which can solve the problem of local boundary image aliasing. The common local deformation algorithm and DBN algorithm are used to process the image for several times, and the comparison curves of the number and accuracy of the two methods are shown in Figure 9. When the graph is unified, the curve of error coefficients of the two algorithms varying with time rate is shown in Figure 10.

As can be seen from the above comparison figure, with the increase of pixels, the ordinary deformation algorithm cannot guarantee that the accuracy changes in a stable state range, and the DBN algorithm can improve the accuracy with the increase of pixels. With the increase of the time rate, the DBN algorithm can reduce the error coefficient to the expected range of the error coefficient, so we suggest using the DBN algorithm to preprocess graphics in information graphics design. The DBN algorithm can improve the accuracy of the model and reduce the error coefficient in graphic design generation.

## 5. Conclusion

With the continuous development of the information society, we begin to pay attention to how to express the meaning of information efficiently and quickly. Many scientific studies show that the deep learning algorithm can train the model and achieve the purpose of information visualization graphic design to spread the message. This paper first analyses the meaning and function of information graphics design and the development trend of the deep belief DBN algorithm in deep learning. According to many research results of the DBN algorithm, the application technology of the DBN algorithm in information visualization graphic design teaching is proposed. Then, the DBN algorithm is studied and discussed in the information graphic design and reconstruction technology, and the adaptive algorithm is introduced in the pretraining stage to find the optimal solution of the output data. The information graphics processed by the DBN algorithm can simplify the original image and form the gray coefficient image. This method can solve the problem of model confusion when a large number of information and graphic data are input. The gray coefficient image is added to the teaching simulation model as the basic data for students to query or reconstruct graphics. The results show that the image reconstruction quality, training speed, and accuracy can be improved in the pretraining and fine-tuning phase of the DBN algorithm. Compared with the traditional algorithm, it has better feasibility and applicability. Finally, the paper studies the technology of the DBN algorithm in information visualization graphic design deformation operation and analyses the results of the DBN algorithm and traditional algorithm in error coefficient, time rate, and accuracy. Experiments show that the DBN algorithm has higher accuracy in processing graphics and can provide a large number of high-quality graphics data for the teaching visualization platform.

## Figures and Tables

**Figure 1:** Deep belief network structure.

**Figure 2:** RBM operation structure diagram.

**Figure 3:** DBN algorithm and performance analysis diagram of the general reconstruction system.

**Figure 4:** Comparison of the feedback speed curve between the quasi-Newton algorithm and BP algorithm in comparison of objective function parameters.

**Figure 5:** Graphic design of deformation after DBN algorithm processing.

**Figure 6:** Comparison curve of the number of feature points between the DBN algorithm processing graph and original graph under clarity.

**Figure 7:** Gray image processed by the DBN algorithm.

**Figure 8:** Comparison of the reconstruction effect between the DBN algorithm and traditional algorithm.

**Figure 9:** Figure pixel number and accuracy comparison curve.

**Figure 10:** Curves of error coefficients of two algorithms varying with the time rate.

## Data Availability

The data used to support the findings of this study are available from the corresponding author upon request.

## References

[1] Goh G., Cammarata N., Voss C. (2021). Multimodal neurons in artificial neural networks. *Distill*.

[2] Abbas A., Sutter D., Zoufal C., Lucchi A., Figalli A., Woerner S. (2021). The power of quantum neural networks. *Nature Computational Science*.

[3] Li X. Z. (2021). A physical layer fusion authentication scheme using deep belief network. *Software Guide*.

[4] Zhong E. D., Bepler T., Berger B., Davis J. H. (2021). CryoDRGN: reconstruction of heterogeneous cryo-EM structures using neural networks. *Nature Methods*.

[5] Samek W., Montavon G., Lapuschkin S., Anders C. J., Muller K.-R. (2021). Explaining deep neural networks and beyond: a review of methods and applications. *Proceedings of the IEEE*.

[6] Hu L., Li Z Z., Ye X. (2020). Delineating and modeling activity space using geotagged social media data. *Cartography and Geographic Information Science*.

[7] Ghorbani B., Mei S., Misiakiewicz T., Montanari A. (2021). Linearized two-layers neural networks in high dimension. *Annals of Statistics*.

[8] Hu X., Che Y., Lin X. (2020). Battery health prediction using fusion-based feature selection and machine learning. *IEEE Transactions on Transportation Electrification*.

[9] Ma M., Sun Y., Fan G. Y. (2021). ECT image reconstruction algorithm based on deep belief network. *Acta Metrologica Sinica*.

[10] Honkura Y., Honkura S. (2020). The development of ASIC type GSR sensor driven by GHz pulse current. *Sensors*.

[11] Mu T., Liu K., Zhou T. (2021). Intelligent diagnosis system of escalator braking force based on deep belief network. *China Elevator*.

[12] Qiao C., Li D., Guo Y. (2021). Evaluation and development of deep neural networks for image super-resolution in optical microscopy. *Nature Methods*.

[13] Shi Y. Y., Pei Z. L., Jiang M. Y. (2021). Review of text classification based on deep belief network. *Journal of Inner Mongolia University for Nationalities*.

[14] Su F., Lu Q., Luo R. Z. (2019). Review of image classification based on deep learning. *Telecommunication science*.

[15] Xiong Z., Lin Y., Li X. (2020). Modelling of 330 MW circulating fluidized bed boiler system based on deep belief network, Journal of Physics: Conference Series. *IOP Publishing*.

[16] Ding M. K., Xu Y. L., Jiang C. J. (2016). Review of deep belief network. *Industrial control computer*.

[17] Yang Y. J. (2020). Teaching reform of graphic design specialty based on information graphic thinking. *Xueyuan*.

[18] Kim J. Z., Lu Z., Nozari E., Pappas G. J., Bassett D. S. (2021). Teaching recurrent neural networks to infer global temporal structure from local examples. *Nature Machine Intelligence*.

[19] Farrell M. H., Liang T., Misra S. (2021). Deep neural networks for estimation and inference. *Econometrica*.

[20] Seeland M., Mäder P. (2021). Multi-view classification with convolutional neural networks. *PLoS One*.

[21] Shi L., Li B., Kim C., Kellnhofer P., Matusik W. (2021). Towards real-time photorealistic 3D holography with deep neural networks. *Nature*.

[22] Liu P. F., Bi J. K., Zhai S. J. (2020). Design and application of intelligent multimedia teaching system. *Modern information technology*.

[23] Xu X. Y. (2020). Research on online teaching practice of multi platform integration. *Computer and information technology*.

[24] Wang X., Gu H., Lu B. (2020). Paradoxical reduction and the bifurcations of neuronal bursting activity modulated by positive self-feedback. *Nonlinear Dynamics*.

[25] Dourado C. M. J. M., da Silva S. P. P., da Nobrega R. V. M., Reboucas Filho P. P., Muhammad K., de Albuquerque V. H. C. (2020). An open IoHT-based deep learning framework for online medical image recognition. *IEEE Journal on Selected Areas in Communications*.

[26] Zhang L., Wang X., Yang D. (2020). Generalizing deep learning for medical image segmentation to unseen domains via deep stacked transformation. *IEEE Transactions on Medical Imaging*.

[27] Guo L.-L., Woźniak M. (2021). An image super-resolution reconstruction method with single frame character based on wavelet neural network in internet of things. *Mobile Networks and Applications*.

[28] Orujov F., Maskeliūnas R., Damaševičius R., Wei W. (2020). Fuzzy based image edge detection algorithm for blood vessel detection in retinal images. *Applied Soft Computing*.

[29] Lopes N., Ribeiro B. (2014). Towards adaptive learning with improved convergence of deep belief networks on graphics processing units. *Pattern Recognition*.

[30] Liu Y., Zhou S., Chen Q. (2011). Discriminative deep belief networks for visual data classification. *Pattern Recognition*.

